# Impact of the First and Second Lockdown for COVID-19 Pandemic on Preterm Birth, Low Birth Weight, Stillbirth, Mode of Labor, and of Delivery in Lombardy, Italy

**DOI:** 10.3390/jpm13030499

**Published:** 2023-03-10

**Authors:** Giovanna Esposito, Marta Rossi, Alessandro Favilli, Matteo Franchi, Giovanni Corrao, Fabio Parazzini, Carlo La Vecchia

**Affiliations:** 1 Department of Clinical Sciences and Community Health, University of Milan, 20122 Milan, Italy; 2 Section of Obstetrics and Gynecology, Department of Medicine and Surgery, University of Perugia, 06156 Perugia, Italy; 3 Unit of Biostatistics, Epidemiology and Public Health, Department of Statistics and Quantitative Methods, University of Milano-Bicocca, 20126 Milan, Italy; 4 National Centre for Healthcare Research and Pharmacoepidemiology, 20126 Milan, Italy

**Keywords:** COVID-19, lockdown, perinatal outcomes, labor, delivery

## Abstract

We investigated the effect of lockdown measures implemented in Lombardy on selected obstetric and perinatal outcomes. Births that occurred during the two lockdowns imposed (i.e., the first from 16 March to 2 June 2020 and the second from 3 November 2020 to 5 April 2021) and the comparison periods (i.e., the first from 16 March to 2 June 2018 and the second from 3 November 2018 to 5 April 2019) were identified using regional healthcare databases. The distribution of births according to the selected outcomes was computed and the Chi-square test was used for testing differences in the periods compared. During the two lockdowns, we observed a lower proportion of low birth weight, from 6.8% in the comparison period to 6.1% in the first lockdown (*p* = 0.019), and from 6.5% to 6.1% in the second one (*p* = 0.109). The proportion of preterm births decreased from 6.8% to 6.3% in the first lockdown (*p* = 0.097), and from 6.2% to 6.0% in the second one (*p* = 0.172). No differences in stillbirth rate emerged for both lockdowns. Induction of labor was more frequent during both lockdowns, from 28.6% to 32.7% in the first (*p* < 0.0001), and from 29.9% to 33.2% in the second one (*p* < 0.0001). Cesarean section was less frequent during the second lockdown.

## 1. Introduction

The COVID-19 pandemic, declared by the World Health Organization (WHO) on 11 March 2020, had largely altered the context of health care. Healthcare systems faced significant challenges responding to the rapid spread of the virus, and radical changes to the way healthcare was delivered were strictly required, thus also suspending deferrable and non-urgent hospitalizations and outpatient services [1].

Changes also impacted on maternity care. Italian hospitals implemented restrictions on visiting in order to minimize contact between people in an effort to combat the transmission of the virus. The restrictions were exacerbated or eased according to the periods of greater or lesser diffusion. Specifically, two lockdown periods, in correspondence with the first and second waves of the pandemic, were imposed.

Several studies from different countries have suggested an impact on perinatal outcomes, such as the timing of delivery and neonatal morbidity and mortality, during national COVID-19 lockdowns. According to a recent review [2], including 17 studies from several countries around the world, lockdown measures were associated with an increased risk of stillbirth with a relative risk (RR) of 1.33 (95% confidence interval (CI): 1.04, 1.69). However, lockdown implementation was not related to a significant risk of preterm birth (PTB) and low birth weight (LBW) compared to pre-pandemic periods. Those data analyzed the impact of the first COVID-19 wave when lockdown measures were generally more stringent.

The evidence regarding the impact of lockdown on the mode of labor and of delivery is not consistent. An analysis of emergency admissions during the first wave of COVID-19 at Clinica Mangiagalli, the largest maternity clinic in Milan, Lombardy, showed a change in the mode of delivery, favoring pre-planned induced births and the hospitalizations for chosen cesarean sections compared to natural births. Most of these changes may be due to the fear of hospital infection that influenced the attitudes of women toward the search for care [3]. However, other studies did not confirm these findings [4].

Although several data have been published on the impact on reproductive outcomes and perinatal assistance during the first wave, less data have been published regarding the impact of the infection during the second wave. The fear of hospital infection was expected to be less marked during the second wave of the COVID-19 pandemic. Further, during the first months of the pandemic, hospitals had implemented more effective organizational measures. Thus, it is conceivable that the impact of the second lockdown was less than that of the first one.

Italy was the first western country to experience a widespread COVID-19 outbreak, and Lombardy, its largest region with about 10,000,000 inhabitants, experienced one of the deadliest COVID-19 outbreaks in the world. In this paper, we analyzed the frequency of selected perinatal outcomes, such as PTB, LBW, stillbirth, mode of labor, and mode of delivery, in Lombardy during the two lockdown periods and compared the results with the corresponding periods of 2018–2019.

## 2. Materials and Methods

### 2.1. Cohort Selection

We retrieved data from the regional healthcare databases of Lombardy, including an archive of demographic and administrative data on all residents who received National Health Service (NHS) assistance. A standard form is used to register all discharges from public or private hospitals (scheda di dimissione ospedaliera (SDO)), and a specific form is filled out at delivery (certificato di assistenza al parto (CedAP)), reporting information about maternal characteristics, pregnancy, and delivery. A deterministic record linkage between the two databases through a unique identification code included in both databases allowed us to identify an unselected birth cohort. Births that occurred in the region during lockdown, due to the COVID-19 pandemic, and the respective comparison periods were identified. Data regarding the COVID-19 infection of pregnant women were not available. We excluded (1) deliveries that did not match to a SDO related to childbirth, (2) deliveries of women aged less than 13 or more than 55, (3) deliveries that did not reach 22 weeks of gestation, and (4) deliveries in which the infant could not be linked to the mother because of a missing identification code.

### 2.2. Definition of Lockdowns and Comparison Periods

In Lombardy, two lockdown periods were imposed by the National and Regional Authorities to face the COVID-19 pandemic: (i) the first from 16 March to 2 June 2020 and (ii) the second from 3 November 2020 to 5 April 2021. Two comparison periods were identified: (i) the first from 16 March to 2 June 2018 and (ii) the second from 3 November 2018 to 5 April 2019.

For the second lockdown period, we chose as a comparison the period from 3 November 2018 to 5 April 2019 because the period from 3 November 2019 to 5 April 2020 overlaps with the first lockdown. Consequently, we considered, also for the first lockdown, the year 2018 as a comparison.

### 2.3. Outcomes of Interest and Data Analysis

We considered selected perinatal outcomes: PTB, LBW, and stillbirth, mode of labor, and mode of delivery. In particular, PTB was defined as any birth before 37 weeks and after 22 weeks of pregnancy [5], and LBW was defined as any child weighing 2500g or less [6].

The distribution of births according to these outcomes during the lockdowns and comparison periods was computed. We presented absolute numbers and percentages. The Chi-square test was used for testing differences regarding the outcomes according to the periods considered.

### 2.4. Ethical Approval

Analysis of an administrative, anonymous database does not require ethical approval in Italy. All data retrieved from the mentioned databases were anonymous.

## 3. Results

A total of 13,476 and 14,952 births were selected during the first lockdown and the comparison period, respectively. During the second lockdown and the comparison period, we identified 25,594 and 29,314 births.

Table 1 provides the distribution of births according to selected perinatal outcomes and mode of labor and delivery during the lockdowns and comparison periods.

The proportion of PTB during the first lockdown period was 6.3% and the corresponding proportion during the same period in 2018 was 6.8% (*p* = 0.097). As for the second lockdown and comparison period, the frequency of PTB was similar (6.0% and 6.2%, respectively; *p* = 0.172).

During the first lockdown, a lower proportion of LBW emerged in comparison to the control period (6.1% vs. 6.8%, *p* = 0.019). However, no differences were observed in the second lockdown (*p* = 0.109).

The stillbirth rate was 3/1000 birth during the first lockdown period and the two comparison periods, and was 2/1000 birth during the second lockdown, without any significant differences.

As regard mode of labor and mode of delivery, induction of labor was more frequent during the first and second lockdowns (*p*-value < 0.0001), while cesarean section was less frequently performed during the second lockdown period (*p* = 0.001) in contrast to the corresponding comparison periods.

## 4. Discussion

In our study, a lower frequency of LBW was observed during the first lockdown period and a lower frequency of PTB also emerged, although not significantly, versus the comparison period. However, no differences were found during the second lockdown. No increase/decrease in stillbirths was observed in either wave of the pandemic. Further, an increase in labor induction was observed in both lockdown periods, and a reduction in cesarean sections was reported during the second one.

Restricted lockdown in Italy was adopted in March–April 2020 when everything, apart from essential activities was closed. In these two months, an excess of over 46,000 deaths was observed in Italy; out of these, over 25,000 were in Lombardy alone. This region was most heavily hit by the first wave in Europe [7,8]. In the second lockdown, lasting from the end of October 2020 to early May 2021, schools and all leisure time activities were closed. However, work was only partly restricted in various regions and in different time periods. The total excess mortality between November 2020 to April 2021 was almost 90,000 deaths in Italy, with a peak of over 25,000 in November 2020 and an attenuated peak in March 2021 [9].

There was an important impact of the COVID-19 pandemic on the Italian healthcare system. In Lombardy, a reduction in recommended healthcare decreased by up to 20% for appropriate gynecologic visits in pregnancy during the first lockdown [10]. Suspending deferrable and non-urgent hospitalizations and outpatient services was not the only result, and the rationing of intensive health resources became a reality in many Italian hospitals [11]. Hospital emergency departments went through a deep reorganization to manage treating critical patients during the pandemic. Inappropriate visits to the emergency departments for non-emergency and low-complexity cases were observed in Lombardy in 2019. However, during the first pandemic wave, also patients in critical condition were reluctant to visit the emergency departments [12].

### 4.1. PTB and LBW

Several studies have reported an impact of the pandemic on PTB and LBW during the period between March and June 2020, although the data are not consistent.

A meta-analysis showed that lockdown was not associated with a PTB risk when compared to the before-lockdown period (RR = 0.93, 95%CI: 0.84–1.03) [2]. Another systematic review confirmed that PTB rates were not significantly changed overall (RR = 0.94, 95%CI: 0.87–1.02), but decreased in high-income countries (RR = 0.91, 95%CI: 0.84–0.99) [4].

A large population study from the Netherlands, which included over 55,000 births that occurred after 9 March 2020, reported a 15–23% decrease in the incidence of PBT in the following months, considering the initial implementation of COVID-19 mitigation measures [13]. In another study from Denmark, the distribution of gestational ages was significantly different (*p* = 0.004) during the lockdown period (12 March to 14 April 2020) compared with the previous 5 years and was driven by a significantly lower rate of extremely premature children [14]. Studies from other European countries, such as Spain [15] and Austria [16], did not confirm these findings. The first did not find any link between prematurity and lockdown and the second one did not observe a significant decrease in late PTB rates. A study from Australia observed an association between lockdown and reduced PTB rates and found that the reduction was stronger in medically indicated than in spontaneous PTB [17]. Similar findings were reported from Africa, specifically in Botswana [18] and in a tertiary care hospital in Arabia [19]. In contrast, data from Israel were inconsistent [20,21].

Within Italy, a study using data from the Lazio hospital discharge database suggested a decrease in the percentage of late PTB in the period March–May 2020 compared to the same period in 2019. There was also an increase, but not a significant one, in very PTB [22]. Another study, covering 10 Italian regions and based on regional health systems, indicated that the pandemic period (1 March to 31 March 2020) compared with the historical one (January 2017 to February 2020) was associated with a reduced risk for PTB (odds ratio (OR) = 0.90; 95%CI: 0.87–0.93) [23].

All the cited studies considered the first wave of infection, but defined lockdown and comparison periods according to different criteria. For this reason, it was not possible to make a consistent comparison across different countries and according to different COVID-19 mitigation measures.

We observed a decreased frequency in PTB only during the first lockdown, but the finding was not significant. Some studies reporting a reduced PTB rate suggested that many of the known risk factors for PTB were affected by the implementation of COVID-19 mitigation measures including lifestyle changes such as cessation of work; increased awareness of hygiene; social distancing; and self-isolation, which resulted in reduction in infections by common pathogens; less physically demanding work; less work-related stress; optimization of sleep duration; and less air pollution [13,14,17].

Only a few studies investigated the weight at birth [15,16], obtaining controversial results. In a meta-analysis, no significant difference associated with the pandemic period was reported in the frequency of LBW (RR = 0.57, 95%CI: 0.24–1.38) on the basis of results from three studies [2].

Our results showed a reduced frequency of LBW during the first lockdown, probably due to the reduction, even if not significant, in PTB in the same period.

### 4.2. Stillbirths

Two meta-analyses reported that lockdown measures during the COVID-19 first wave were associated with about a 30% increased risk of stillbirth [2,4]. Studies from different countries are, however, controversial. Data from the United Kingdom [24] reported that stillbirths increased, with a difference of 6.93/1000 births (95%CI 1.83, 12.0) when comparing the period 1 February 2020 to 14 June 2020 and 1 October 2019 to 1 January 2020. Likewise, in an Italian study, a nearly threefold increase in stillbirths was observed when the stillbirth rate went from 10 to 26 per 1000 total births between 2019 and 2020 (March to May) [22]. Conversely, an Australian investigation found a decrease in stillbirth rates during lockdown [17].

According to an Italian study conducted in Milano, five fetal deaths were diagnosed at emergency services from 23 February to 23 June 2020, in comparison with one fetal death observed in the same period in 2019 (*p* = 0.04). Authors suggested that the lockdown negatively influenced emergency service admissions and, consequently, the women’s reproductive health, and hypothesized that the women were inclined to wait longer for a visit due to the fear of in-hospital contagion [3].

However, other studies from Spain [15] and from the United States [25] found no significant differences in stillbirth rates before and during the pandemic. Again, a recent analysis of the Bavarian perinatal data showed that during the first lockdown, the stillbirth rate was significantly higher compared to previous years. However, the finding was not significant after adjustment for seasonal and long-term trends. During the second lockdown, the stillbirth rate did not differ compared to the years from 2010 to 2019 [26]. No increase in the stillbirth rate was also observed in the previously cited Italian study on several regions when comparing the first wave period with previous years (up to 2017) [23].

We confirmed these findings. In particular, no increase in the stillbirth rate was observed during the two lockdown periods considered.

### 4.3. Mode of Labor and Delivery

Data regarding the mode of labor and delivery during the pandemic are scarce.

As for the mode of labor, the previously quoted systematic review observed an increase in induction of labor in Nepal, the only low-middle-income country included (OR = 2.26, 95%CI 2.12–2.42) [27], but reported an absence of association between lockdown and induction of labor in high-income countries (OR = 1.15, 95%CI 0.81–1.64) [4].

However, the data from different studies were inconsistent. According to an Italian study, the frequency of elective caesarean section and labor induction increased, respectively, from 20% and 27% in 2019 to 23% and 30% in 2020 (*p* = 0.014). This increase was attributable to the fear that the hospital stay may increase the risk of COVID-19 infection [3]. In contrast, a study from the United States, aimed at evaluating the length of stay in the hospital after the birth, found that there was no difference in induction of labor and cesarean delivery rates [28].

An Italian study suggested a non-significant reduction in caesarean sections [22]. A study focusing on changes in the indications for cesarean delivery after the lockdown in Wuhan found that cesarean section on maternal request and fetal distress was significantly more common in the group of women who delivered during the first COVID-19 wave than in a comparison period [29].

In our cohort, we observed an increased frequency in labor induction in both the lockdown periods and a reduction in cesarean sections during the second one.

### 4.4. Limitations and Strengths

The lack of information regarding the contagion of women is a limitation of the present work since this did not allow us to distinguish the possible effect of the infection from the impact of the restriction measures on perinatal outcomes, in particular on PTB and LBW. Among the strengths of this study are the large sample sizes and the coverage of the entire period affected by the COVID-19 pandemic. Lombardy is one of the most populous regions of Italy and has been particularly affected by COVID-19 in both the period of the two waves and was the first region outside of Wuhan to be overwhelmed by the pandemic. A specific interest of this analysis was comparing the outcome during the first and second waves. This comparison may provide relevant information regarding the impact of COVID-19 on pregnant women’s healthcare and the effects of the reorganization of health services implemented during the summer of 2020 on clinical practice and reproductive outcomes.

## 5. Conclusions

Our investigation shows that the COVID-19 pandemic and the consequent reorganization of health services implemented had an impact on the management of birth, in particular, resulting in a higher number of labor inductions but a minor impact on maternal and neonatal outcomes. Further efforts are needed to clarify the clinical and organizational reasons underlying these changes.

## Figures and Tables

**Table 1:** The distribution of births according to selected perinatal outcomes, mode of labor, and mode of delivery during lockdowns and comparison periods.

	First Lockdown	Comparison Period		Second Lockdown	Comparison Period	
	16 March to 2 June 2020 (N = 13,476)	16 March to 2 June 2018 (N = 14,952)		3 November 2020 to 5 April 2021 (N = 25,594)	3 November 2018 to 5 April 2019 (N = 29,314)	
	N (%)	N (%)	*p*-Value	N (%)	N (%)	*p*-Value
**Preterm birth**						
No	12,627 (93.7)	13,937 (93.2)	0.097	24,044 (94.0)	27,456 (93.8)	0.172
Yes	849 (6.3)	1015 (6.8)		1550 (6.0)	1858 (6.2)	
**Low birth weight**						
No	12,652 (93.9)	13,935 (93.2)	0.019	24,023 (93.9)	27,417 (93.5)	0.109
Yes	824 (6.1)	1017 (6.8)		1571 (6.1)	1897 (6.5)	
**Stillbirth** ^a^						
No	13,434 (99.7)	14,902 (99.7)	0.525	25,522 (99.8)	29,222 (99.7)	0.074
Yes	41 (0.3)	50 (0.3)		62 (0.2)	92 (0.3)	
**Mode of labor** ^b^						
Spontaneous	7494 (67.3)	8851 (71.4)	<0.0001	14,246 (66.8)	16,964 (70.1)	<0.0001
Inducted	3642 (32.7)	3538 (28.6)		7074 (33.2)	7231 (29.9)	
**Mode of delivery** ^c^						
Vaginal delivery	9983 (76.1)	11,048 (76.0)	0.448	19,083 (76.8)	21,508 (75.5)	0.001
Elective CS	1996 (15.2)	2164 (14.9)		3546 (14.3)	4331 (15.2)	
Urgency CS	1147 (8.7)	1326 (9.1)		2212 (8.9)	2665 (9.3)	

^a^ The sum did not add up to the total because of missing data (1 (less than 0.1%) in the group of first lockdown period and 10 (less than 0.1%) in the group of second lockdown period). ^b^ The sum did not add up to the total because of missing data (2 (less than 0.1%) in the group of the first comparison period, 2 (less than 0.1%) in the group of the second lockdown period, and 5 (less than 0.1%) in the group of the second comparison period) and the exclusion of deliveries with no labor (2340 (17.4%) in the group of first lockdown period, 2561 (17.1%) in the group of first comparison period, 4272 (16.7%) in the group of second lockdown period, and 5114 (17.5%) in the group of second comparison period). ^c^ The sum did not add up to the total because of missing data (350 (2.6%) in the group of first lockdown period, 414 (2.8%) in the group of first comparison period, 753 (2.9%) in the group of second lockdown period, and 810 (2.8%) in the group of second comparison period).

## Data Availability

The data that support the findings of this study are available from Lombardy Region, but restrictions apply to the availability of these data, which were used under license for the current study. The data used in this study cannot be made available in the manuscript, or in a public repository due to Italian data protection laws. The anonymized datasets generated during and/or analyzed during the current study can be provided on reasonable request, from the corresponding author, after written approval by the Lombardy region.
